# Prediction of intraperitoneal adhesions using striae gravidarum and scar characteristics in women undergoing repeated cesarean sections

**DOI:** 10.1186/s12884-021-03763-z

**Published:** 2021-04-09

**Authors:** Mohamed Elprince, Omima T. Taha, Zakia M. Ibrahim, Rasha E. Khamees, Mahmoud A. Greash, Khaled A. Atwa, Ahmed M. Gadallah, Noha al-Okda, Radwa M. Abdel Aal, Mohamed F. Ibrahim, Ahmed A. Aboelroose, Osama E. Ashour, Asmaa M. Elgedawy, Amira M. Elbahie, Hanan M. Ghoneim, Amal A. Ahmed

**Affiliations:** Department of Obstetrics and Gynecology, Faculty of Medicine, Suez Canal University, Ismailia, Egypt

**Keywords:** Adhesions, Cesarean scar, Prediction, Striae

## Abstract

**Background:**

The current fact of increasing rates of cesarean deliveries is a catastrophe. Recurrent cesareans result in intraperitoneal adhesions that would lead to maternal morbidity during delivery. Great efforts are directed towards the prediction of intraperitoneal adhesions to provide the best care for laboring women. The aim of the current study was to evaluate the role of abdominal striae and cesarean scar characters in the prediction of intraperitoneal adhesions.

**Methods:**

This was a case- control study conducted in the emergency ward of the obstetrics and gynecology department of a tertiary hospital from June to December 2019. The study was carried on patients admitted to the ward fulfilling particular inclusion and exclusion criteria. The study included two groups, group one was assessed for the presence of striae, and the degree of intraperitoneal adhesions was evaluated during the current cesarean section. Group two included patients without evidence of abdominal striae. They were evaluated for the severity of adhesions also after evaluation of the previous scar. Evaluation of the striae was done using Davey’s scoring system. The scar was assessed using the Vancouver Scar Scale. The modified Nair’s scoring system was used to evaluate intraperitoneal adhesions.

**Results:**

The study group included 203 women, while the control group included 205 women. There were significant differences in the demographic characters of the recruited patients (*p*-value 0.001 for almost all variables). The mean Davey score in those with mild, moderate, and severe striae was 1.82 ± 0.39, 3.57 ± 0.5, and 6.73 ± 0.94, respectively (p-value < 0.001). Higher scores for the parameters of the Vancouver scale were present in patients with severe striae (1.69 ± 1.01, 1.73 ± 0.57, 2.67 ± 1.23, and 1.35 ± 1.06 for scar vascularity, pigmentation, pliability, and height respectively with a p-value of < 0.001 each). Thick intraperitoneal adhesions were noted significantly in women with severe striae [21 (43.75%), *p*-value < 0.001)]. The Davey’s and Vancouver scores showed highly significant predictive performance in the prediction of intraperitoneal adhesions (*p*-value < 0.001).

**Conclusion:**

Abdominal striae and cesarean scar were significant predictors for intraperitoneal adhesions.

## Background

Intra-abdominal adhesions contribute significantly to surgical morbidity in addition to infertility. Cesarean section (CS) is considered one of the most commonly practiced surgical procedure by obstetricians. This raised the assumption that the prediction of intraabdominal adhesions would lead to decreased morbidity [1]. Intraabdominal adhesions occur at a 7% rate after one CS up to 68% with repeated cesareans [2].

Striae are linear skin changes in areas of skin stretching that cause bothering disfigurement. This occurs because of dermal damage. This stretching occurs due to pregnancy, as well as obesity and Cushing syndrome [3]. By examination, they appear as pink– purple and, finally, depressed white lines. Histologically, these areas are characterized by a decreased extracellular matrix as well as decreased collagen [4].

The epidermis at the site of the abdominal scars demonstrates delicate well-organized collagen bundles arranged parallel to each other [5]. However, scars do not heal similarly, raising the suggestion of a possible relationship to intra-abdominal adhesions [6].

The similarity in the formation of these changes raised the possibility of using abdominal striae and scar appearance as predictive tools for the severity of intra-abdominal adhesions. Because of the conflicting results about the role of abdominal striae and cesarean scar characters in the prediction of intra- abdominal adhesions [7–12], the current study was conducted.

## Methods

This study was conducted as a case control study after approval of the research ethics committee of the faculty of medicine, Suez Canal University, in May 2019 with a number of 3849. We recruited patients over six months. The study was carried out in the obstetrics and gynecology department, Suez Canal University Hospitals.

The study was carried on patients admitted to the ward fulfilling the following inclusion and exclusion criteria. Inclusion criteria: - a) patients with previous CS, b) patients presenting for emergency or elective CS delivery. Exclusion criteria: - a) previous midline surgery, b) history of wound complications, c) history of endometriosis, d) history of pelvic inflammatory disease (PID), e) other abdominal operations other than CS, f) keloid scar formation, g) chronic steroid therapy, h) Cushing disease, i) adrenal hyperplasia, j) Ehlers-Danlos syndrome, k) Marfan syndrome, l) Skin disease as lichen sclerosis, m) Prolonged progesterone use, n) history of multiple pregnancies, o) history of hydramnios, p) history of macrosomic babies and q) family history of striae on other parts of the body (breast, hips, and buttocks).

After fulfilling the above criteria, the study included two groups. Group one was assessed for the presence of striae and the degree of intra-abdominal adhesions was evaluated during the current CS. Group two included patients without evidence of abdominal striae and were evaluated for the severity of adhesions after evaluating the previous scar.

All participants gave written informed consent before entering the study. Patients eligible for the study had the following:-

a- Preoperative evaluation: including personal data (age, weight, height, BMI, occupation, level of education, contact information), obstetric history (parity, gestational age, number of previous CS), and any chronic illness. A blood sample for a group and save was withdrawn.
b- Evaluation of striae: using Davey’s scoring system [13]. In this system, the abdomen is divided into four quadrants using vertical and horizontal lines passing by the umbilicus. Each quadrant is examined for the striae and scored in the following manner:

1. Clear skin, scored as 0
2. A moderate number of striae scored as 1
3. Many striae, scored as 2.

This leads to a total score of 0–8. The severity of striae is classified as none (0), mild [1, 2], moderate [3, 4], or severe [5–8]. Evaluation of the striae was done by the same researcher using the figure provided by Buchanan et al. [13]. Evaluation of intraabdominal adhesions was done by another researcher. Both of them were blinded to the results reported by each other.

c- The scar was assessed using the Vancouver Scar Scale (VSS). This scale evaluates the scar for pigmentation, vascularity, pliability, and height [14].
d- Intraperitoneal adhesions were evaluated by the modified Nair’s scoring system. This system classified adhesions into no adhesions, thin filmy adhesions (either single or two bands of adhesions between viscera or from viscera to the abdominal wall), and thick, dense adhesions (more than two bands between viscera or from viscera to the abdominal wall, multiple dense adhesions, or viscera directly adherent to the abdominal wall, regardless of the number or extent of the bands) [15].

Striae and scare characters were evaluated by a researcher who was blinded to the extent of intraperitoneal adhesions.

### Statistical analysis

Data were statistically described in terms of mean and standard deviation, frequencies (number of cases), and percentages when appropriate. *P* values less than 0.05 were considered statistically significant. All statistical calculations were done using computer program SPSS (Statistical Package for the Social Science; SPSS Inc., Chicago, IL, USA) release 22 for Microsoft Windows. Chi-square test was used for categorical variables and (t) test for continuous variables with normally distributed data. Non-normally distributed data were tested using non-parametric tests. Receiver operator characteristic curve was constructed for the Davey’s and Vancouver scores to have its cutoff point for the prediction of intraperitoneal adhesions. Sensitivity and specificity were calculated. For the construction of logistic regression models for the prediction of intraperitoneal adhesions, the dependent variable was the presence or absence of adhesions. This was put against all of the variables that it depended upon; hence, there were multiple simple logistic models each with a significant factor. These significant factors were put in a model and factors were removed one by one to produce a best-fit multiple logistic model.

## Results

We recruited patients over six months from June to December 2019. The study group included 203 women, while the control group included 205 women. Data were analyzed according to the grade of Davey’s score (mild, moderate, and severe). Patients with no evidence of abdominal striae were considered as controls. Subgroup analysis of the study group was done according to the severity of their Davey’s’ score. There were significant differences in the demographic characters of the recruited patients (*p*-value 0.001 for almost all variables) (Table 1).

**Table 1:** Patient demographic data according to the distribution of abdominal striae

Davey’s score grade	None	Mild	Moderate	Severe	*p*-value
**Age (years) (Mean ± SD)**	27.92 ± 3.1	29.5 ± 5.76	31.96 ± 5.67	33.23 ± 4.68	***< 0.001***
**Parity (Mean ± SD)**	1.28 ± 0.45	2.17 ± 1.31	2.57 ± 1.53	2.75 ± 1.55	***< 0.001***
**Number of previous CS (Mean ± SD)**	1.22 ± 0.42	1.72 ± 0.85	1.87 ± 0.91	2.52 ± 1.38	***< 0.001***
**Weight (kg) (Mean ± SD)**	76.46 ± 11.66	80.14 ± 10.55	86.22 ± 11.05	84.38 ± 13.49	***< 0.001***
**Height (cm) (Mean ± SD)**	164.98 ± 6.92	162.62 ± 5.38	162.96 ± 5.58	164.71 ± 4.27	***< 0.001***
**Body mass index (kg/m^2) (Mean ± SD)**	28.11 ± 4.2	30.41 ± 4.47	32.52 ± 4.21	31.05 ± 4.67	***< 0.001***

The mean Davey score in those with mild, moderate, and severe striae was 1.82 ± 0.39, 3.57 ± 0.5, and 6.73 ± 0.94, respectively (*p*-value < 0.001). Higher scores for the parameters of the Vancouver scale were present in patients with severe striae (1.69 ± 1.01, 1.73 ± 0.57, 2.67 ± 1.23, and 1.35 ± 1.06 for scar vascularity, pigmentation, pliability, and height respectively with a *p*-value of < 0.001 each). Thick intraperitoneal adhesions were noted significantly in women with severe striae [21 (43.75%), *p*-value < 0.001) (Table 2).

**Table 2:** Scare characters and intrabdominal adhesions in relation to abdominal striae

Davey’s score grade		None (205)	Mild (109)	Moderate (46)	Severe (48)	*p*-value
**Vascularity (Mean ± SD)**		0.61 ± 0.82	0.89 ± 0.64	1.07 ± 0.8	1.69 ± 1.01	***< 0.001***
**Pigmentation (Mean ± SD)**		0.84 ± 0.83	1.01 ± 0.73	1.54 ± 0.62	1.73 ± 0.57	***< 0.001***
**Pliability (Mean ± SD)**		1.11 ± 0.99	1.34 ± 1.05	1.83 ± 1.34	2.67 ± 1.23	***< 0.001***
**Height (mm) (Mean ± SD)**		0.56 ± 0.76	0.77 ± 0.73	1 ± 0.89	1.35 ± 1.06	***< 0.001***
**Total score (/13) (Mean ± SD)**		3.12 ± 2.97	4.01 ± 2.52	5.43 ± 2.75	7.44 ± 2.92	***< 0.001***
**Davey’s score (Mean ± SD)**		0 ± 0	1.82 ± 0.39	3.57 ± 0.5	6.73 ± 0.94	***< 0.001***
**Intraperitoneal adhesions (N%)**	**None**	171 (83.41%)	24 (22.02%)	9 (19.57)	10 (20.83)	***< 0.001***
	**Thin filmy**	34 (16.59%)	74 (67.89%)	24 (52.17)	17 (35.42)	
	**Thick**	0 (0%)	11 (10.09%)	13 (28.26)	21 (43.75)	

Women with intraperitoneal adhesions had more vascular, hyperpigmented, less liable, and elevated scars than those without (*p*-value < 0.001 each) (Table 3).

**Table 3:** Scar characters in women with intraperitoneal adhesions

Adhesion occurrence		No	Yes	*p*-value
Variable	Attribute	n (%)	n (%)	
**Vascularity**	**Normal**	127 (59.35)	32 (16.49)	***< 0.001***
	**Red**	57 (26.64)	114 (58.76)	
	**Pink**	14 (6.54)	38 (19.59)	
	**Purple**	16 (7.48)	10 (5.15)	
	**Total**	214 (100)	194 (100)	
**Pigmentation**	**Normal**	96 (44.86)	28 (14.43)	***< 0.001***
	**Hypopigmented**	44 (20.56)	88 (45.36)	
	**Hyperpigmented**	74 (34.58)	78 (40.21)	
	**Total**	214 (100)	194 (100)	
**Pliability**	**Normal**	66 (30.84)	16 (8.25)	***< 0.001***
	**Supple**	90 (42.06)	83 (42.78)	
	**Yielding**	47 (21.96)	36 (18.56)	
	**Firm**	0 (0)	42 (21.65)	
	**Ropes**	11 (5.14)	8 (4.12)	
	**Contracture**	0 (0)	9 (4.64)	
	**Total**	214 (100)	194 (100)	
**Height (mm)**		0.5 ± 0.75	1.05 ± 0.85	***< 0.001***
**Total score (/13)**		3.08 ± 3.08	5.28 ± 2.81	***< 0.001***

The Davey’s and Vancouver scores showed highly significant predictive performance in the prediction of intraperitoneal adhesions (*p*-value < 0.001) (Table 4).

**Table 4:** Linear regression model for the prediction of intra-peritoneal adhesions

Variables	β	*P*-value	OR	95% CI OR
**Age (years)**	0.217	***< 0.001***	1.243	(1.156–1.335)
**Education**	−2.093	***< 0.001***	0.123	(0.071–0.215)
**Body mass index**	0.083	***0.008***	1.086	(1.022–1.155)
**Vancouver score**	0.236	***< 0.001***	1.267	(1.119–1.433)
**Davey score**	0.479	***< 0.001***	1.615	(1.374–1.898)

Davey’s score of ≥1 significantly predicted intraperitoneal adhesions with a sensitivity and specificity of 82.47 and 79.91%, respectively. Also, a Vancouver score of 2 was highly significant in the prediction of intraperitoneal adhesions. It had a sensitivity of 84.02% and specificity of 56.07% (Table 5, Fig. 1).

**Table 5:** Cut- off value for the Davey score and the Vancouver score

Variable	AUC	*p*-value	Cut-off point	Sensitivity	Specificity	PPV	NPV	LR+	LR-
Davey’s score	0.811	***< 0.001***	1	82.47	79.91	78.8	83.4	4.1	0.22
Vancouver score	0.719	***< 0.001***	2	84.02	56.07	63.4	79.5	1.91	0.28

**Fig. 1:** ROC (Receiver Operating Characteristics) curve showing the diagnostic accuracy of the Davey’s and Vancouver’s scores in the prediction of intra-abdominal adhesions

## Discussion

Nearly half of the studied population had abdominal striae. There were discrepancies in the prevalence of abdominal striae in the previous studies with rates of 65.7, 67.7% among Egyptian women [7, 16] and 80, and 57.9% among Turkish women [8, 17]. This would be rendered to different sample sizes as well as different races among the studied populations.

The subanalysis performed for the study group demonstrated significant differences in the demographic characters. In the cohort evaluated in a recent study, there were no differences in the demographic data of the recruited population [7]. However, in the cohort evaluated by another researcher, a significant difference was reported between the three groups in age, BMI, weight gain during pregnancy, and fetal weight [16]. Such differences would be rendered to different patient grouping (no/mild striae as a group and severe striae as the other one in the former, and no, mild and severe striae in the latter).

Thick intraperitoneal adhesions were noted significantly in women with severe striae. This was following the results reported by Abbas et al.; however, they reported that 90% of women with severe striae had thick adhesions with mean Davey score of 4.25 ± 3.36 [7]. Another study reported close results to the current one (50% of patients with severe striae had dense adhesions) [8]. This difference would be explained by the different samples included besides; both studies divided patients into two groups only.

In contention with the current study, there was no difference in peritoneal adhesions in women with or without striae [9, 10]. However, another study reported higher rates of intraperitoneal adhesions in women with no or mild striae than those with severe striae (67.3, 65.9, and 36.3%, respectively) [17]. This was explained by the frequent presence of dysfunctional fibroblasts in striae and adhesions. Fibroblasts have an essential role in collagen production in the adhesions; accordingly adhesion formation decreases [17]. Besides, the different tools for evaluation of the striae would result in variable results, especially when incorporating the striae color, which was not evaluated in the current study.

The current study reported intraperitoneal adhesions occurring in 194/ 408 (47.5%) of the studied population. This was lower than reported by others (59.6 and 54.3%) [16, 17]. However, too much higher rates of intraperitoneal adhesions were reported by Abbas et al. and Khalifi et al. (87 and 73.5%, respectively) [7, 18]. This disparity in results would be rendered to differences in surgeons, techniques, and suture materials used in the operations.

Women with severe striae and those with intraperitoneal adhesions had more vascularized, hyperpigmented, less pliable and elevated CS scars. This contradicted the results reported by previous research, which stated that flat unpigmented scars were more prominent in women with striae. They explained this by the overexpression of transforming growth factor- Beta. It leads to deficient elastin production, which is a causative factor in the formation of abdominal striae [9].

To achieve perfect scar remodeling, collagen fibers are organized in a parallel fashion. While, in elevated scars, increased collagen production is noted. This was thought to arise from variability in transforming growth factor-beta, which plays an essential role in the formation of hypertrophic scars as well as intraperitoneal adhesions [17]. Scar width and appearance showed significant association with dense intraperitoneal adhesions (*p*-value 0.001, and 0.002 respectively) [10]. Depressed hypopigmented scars were also associated with adhesions, which were assumed to arise from the inward traction from the adhesion bands [19, 20]. Besides, in a meta-analysis of numerous studies, they reported that flat scars were indicative of absent adhesions while depressed ones were associated with adhesions [11]. Conflicting results exist as elevated scars were found to be associated with more adhesions all over the abdomen than flat or depressed ones [12].

The Davey’s and Vancouver scores showed a highly significant predictive performance in the prediction of intraperitoneal adhesions. This was similar to the results reported previously, where Davey score of 2 was considered a significant risk factor in predicting intraperitoneal adhesions. Also, the best cut off was ≥3 with reported sensitivity and specificity of 64 and 51.3%, respectively [7] with higher results reported by the current study at a cut off ≥1. However, Abdelaal et al. reported that abdominal striae were not considered a predictor for abdominal adhesions while the number of previous CS did [16].

### Research implications

The role of the scar characters in relation to intraperitoneal adhesions needs to be evaluated deeply. Further studies evaluating the impact of intra- abdominal adhesions on the difficulty of the cesarean delivery are recommended. This would be represented by the total duration of the operation, need for blood transfusion, and possible visceral injury.

## Strengths and limitations of the study

Strengths included a large sample size of recruited patients; subanalysis of the patients with striae into mild, moderate and severe provided more robust results, evaluation of the striae and CS scar using simple scoring systems, and the recruited population was of the same ethnicity. However, we did not have any previous medical records about the operative notes of the previous deliveries since most of them delivered in private sittings outside the hospital previously. We did not consider the inter-pregnancy interval as a risk factor for adhesion formation. Also, we did not evaluate the color of the striae. We did not evaluate the impact of the dense adhesions on the difficulty of the cesarean delivery.

## Conclusion

Abdominal striae and CS scar were significant predictors for intraperitoneal adhesions. Women with severe striae had thick intraperitoneal adhesions. Women with intraperitoneal adhesions had more vascular, hyperpigmented, less pliable and elevated scars.

## Data Availability

The datasets used and/or analyzed during the current study available from the corresponding author on reasonable request. All data generated or analyzed during this study are included in this published article.

## Abbreviations

CS: Cesarean section
PID: Pelvic inflammatory disease
BMI: Body mass index
VSS: Vancouver Scar Scale
